# Production and characterization of a biosurfactant produced by *Streptomyces sp*. DPUA 1559 isolated from lichens of the Amazon region

**DOI:** 10.1590/1414-431X20176657

**Published:** 2017-12-11

**Authors:** A.P.P. Santos, M.D.S. Silva, E.V.L. Costa, R.D. Rufino, V.A. Santos, C.S. Ramos, L.A. Sarubbo, A.L.F. Porto

**Affiliations:** 1 Departamento de Morfologia e Fisiologia Animal, Universidade Federal Rural de Pernambuco, Recife, PE, Brasil; 2 Departamento de Química, Universidade Federal Rural de Pernambuco, Recife, PE, Brasil; 3 Centro de Ciências e Tecnologia, Universidade Católica de Pernambuco, Recife, PE, Brasil

**Keywords:** Biosurfactant, Surface tension, Emulsification, Streptomyces, Soybean frying oil

## Abstract

Surfactants are amphipathic compounds containing both hydrophilic and hydrophobic groups, capable to lower the surface or interfacial tension. Considering the advantages of the use of biosurfactants produced by microorganisms, the aim of this paper was to develop and characterize a biosurfactant produced by *Streptomyces sp.* DPUA1559 isolated from lichens of the Amazon region. The microorganism was cultured in a mineral medium containing 1% residual frying soybean oil as the carbon source. The kinetics of biosurfactant production was accompanied by reducing the surface tension of the culture medium from 60 to values around 27.14 mN/m, and by the emulsification index, which showed the efficiency of the biosurfactant as an emulsifier of hydrophobic compounds. The yield of the isolated biosurfactant was 1.74 g/L, in addition to the excellent capability of reducing the surface tension (25.34 mN/m), as observed from the central composite rotational design when the biosurfactant was produced at pH 8.5 at 28°C. The critical micelle concentration of the biosurfactant was determined as 0.01 g/mL. The biosurfactant showed thermal and pH stability regarding the surface tension reduction, and tolerance under high salt concentrations. The isolated biosurfactant showed no toxicity to the micro-crustacean *Artemia salina*, and to the seeds of lettuce (*Lactuca sativa L.*) and cabbage (*Brassica oleracea L*.). The biochemistry characterization of the biosurfactant showed a single protein band, an acid character and a molecular weight around 14.3 kDa, suggesting its glycoproteic nature. The results are promising for the industrial application of this new biosurfactant.

## Introduction

Surfactants are substances widely utilized for cleaning in general, removing undesirable particles or dirtiness by a process called emulsification. Surfactants are amphipathic compounds, containing both hydrophilic (polar) and hydrophobic (nonpolar) groups, capable to lower the surface or interfacial tension between two liquid phases such as oil/water, or air/liquid interfaces (1–3). One of the surfactants widely used in personal care products is the sodium lauryl sulfate. This anionic surfactant is synthesized by reacting lauryl alcohol from a petroleum or plant source with sulfur trioxide (4). The surfactants of biological origin produced by microorganisms (bacteria, yeasts and fungi) are known as biosurfactants (2). The biosurfactants can also be produced by animals; for instance, the type II alveolar epithelial cells (pneumocytes) can synthesize a surface-active phospholipoprotein which is the pulmonary surfactant (5). Biosurfactants are classified based on their chemical structures that include glycolipids, lipopeptides, polysaccharide-protein complexes, phospholipids, fatty acids and neutral lipids (3). Moreover, surfactants can be classified according to the ionization state in aqueous solution as anionic (functional group with negative charge), cationic (functional group with positive charge), nonionic (no charge that influences the aqueous medium, so they do not ionize in aqueous solution) and amphoteric (anionic and cationic characteristic) (6).

In addition to the surface-active properties, biosurfactants produced by some microorganisms have exhibited antimicrobial activity and anti-adhesive activity against several other microorganisms (3,7).

The biosurfactants have attracted attention because of their low toxicity, biodegradability, and ecological acceptability; furthermore, low cost raw materials, such as agricultural and industrial waste can be used as substrates to the biosurfactant production (1).

The properties of biosurfactants allow their utility in various areas of applications such as bioremediation, biodegradation, enhanced oil recovery, pharmaceutics, food processing among many others (7,8).

Over the last few years, species of the genus *Streptomyces* have been used to produce biosurfactants, especially the bacteria of the Actinomycetes group. These bacteria have a filamentous organization, are aerobic, catalase-positive and can inhabit the soil. They are microorganisms of interest for medical, agricultural and biotechnology areas, since most of the strains synthesize antibacterial, antifungal, antitumor, antiparasitic substances, herbicides and enzymes (7,9,10).

Considering the advantages of biosurfactants produced by microorganisms, the aim of this paper was to perform the production and the characterization of a new biosurfactant produced by *Streptomyces sp.* DPUA1559 isolated from lichens of the Amazon region.

## Material and Methods

### Bacterial strain and preparation of seed culture

A strain of *Streptomyces sp* DPUA1559 isolated from lichens of the Amazon region, belonging to the collection of the Departamento de Parasitologia, Universidade Federal do Amazonas (Manaus, AM, Brazil) was used. Sporulated cultures were obtained in Petri dishes with ISP-2 solid medium. The medium was composed of 0.4% (v/v) yeast extract, 1% (v/v) malt extract and 2% (v/v) agar, pH 7.0, and it was incubated in a bacteriological incubator for 15 days at 30°C. The stock culture was kept in cryotubes with 10% (v/v) glycerol, under cooling at –18°C. The microorganism was activated in ISP-2 medium, modified by the absence of glucose according to Pridham et al. (11). The inoculum was obtained after culture in 1.0% (v/v) malt extract and 0.4% (v/v) yeast extract. The pH of the medium was adjusted to 7.0 with 1M NaOH, and it was fermented on an orbital shaker (B. Braun Melsungen AG) under 150 rpm at 28°C for 48 h.

### Fermentation medium and biosurfactant production

Soybean frying oil was used as the carbon source to produce the biosurfactant. The fermentation medium consisted of 10 g/L soybean residual oil, 10 g/L 1% peptone, 4.75 g/L K_2_HPO_4_, 1 g/L NH_4_Cl, 6 g/L MgSO_4_.7H_2_O, and 1 mL of nutrient solution (100 mg FeSO_4_·7H_2_O, 100 mg MnCl_2_·4H_2_O, 100 mg ZnSO_4_·H_2_O, and 100 mg of CaCl_2_·H_2_O), adjusted to pH 7.5 with a solution of 1M NaOH.

The biosurfactant production was conducted in Erlenmeyer flasks (250 mL) containing 50 mL of the fermentation medium inoculated with 108 CFU/mL aliquots of each conical spore in an orbital shaker (B. Braun Melsungen AG) at 200 rpm, 28°C for 96 h.

### Experimental design through central composite rotatable design (CCRD)

A CCRD was used to determine the effects and interactions of two factors for biosurfactant production by *Streptomyces sp.* DPUA1559. Temperature and pH were the independent variables. Surface tension was the response variable. In this design, a set of 12 experiments was performed, with four replicates at the central points. The statistical analysis of the four replicates gives an indication of the experimental error of the production technique. The range and levels of the components (factors or independent variables) are given in Table 1. Each factor in the design was studied on five levels (−1.41, −1.0, 0, +1, and +1.41), with zero as the central coded value. Analysis of variance (ANOVA) with 95% confidence intervals was used to determine the significance of the effects. ANOVA, the determination of regression coefficients and the construction of graphs were performed with the aid of the Statistica^®^ program, version 12.0 (USA).

**Table 1.** Real and coded values of the variables for the central composite rotational design.

Factors	−1.41	−1	0	1	1.41
pH	8.36	8.4	8.5	8.6	8.64
Temperature °C	26.6	27.0	28.0	29.0	29.4

pH: (X_1_); Temperature °C: (X_2_).

### Growth kinetics and biosurfactant production

To determine the growth kinetics, samples were collected every 4 h during the first 12 h, then every 12 h until 120 h of fermentation. The samples were subjected to biomass analysis, determination of pH, surface tension and emulsification index measurements.

### Biomass determination

For biomass determination, 10 mL samples were centrifuged at 5000 *g* for 30 min at 5°C and the cell pellet was dried in an oven at 105°C for 24 h.

### Isolation of biosurfactant

The biosurfactant was extracted from culture media after cell removal by centrifugation at 5000 *g* for 30 min at 5°C. The supernatant pH was adjusted to 2.0 with 6.0 M HCl, and an equal volume of CHCl_3_/CH_3_OH (2:1) was added. The mixture was vigorously shaken for 15 min and allowed to set until phase separation according to Javaheri et al. (12). After phase separation, the concentrate was centrifuged at 3000 *g* for 5 min at 5°C and suspended in Milli-Q water. Then the concentrate was added to a sterile petri dish and neutralized with 1 M NaOH solution to pH 7.0. It was then preserved in a drying oven at 37°C for 12 h. The yield of biosurfactant was obtained in g/L and used to measure the critical micelle concentration (CMC).

### Emulsification index with different hydrophobic compounds

The rate of emulsification was measured using the method described by Cooper and Goldenberg (13). The cell-free fermentation broth was mixed to one of the following hydrophobic compounds (in ratio 1:1, v/v): kerosene, motor oil, residual motor oil, diesel oil, corn oil, canola oil, soybean oil or sunflower oil. The mixture was homogenized in a vortex for 2 min at room temperature. The emulsion stability was determined after 24 h. The emulsification index was calculated as the ratio between the height of emulsifying layer and the total height, being the value obtained multiplied by 100.

### Stability studies

The effect of environmental factors on biosurfactant activity was determined according to Rufino et al. (8). The effect of addition of different concentrations of NaCl on the activity of the biosurfactant was investigated in the cell-free broth. A specific concentration of NaCl (2–10%, w/v) was added and surface tension was determined as previously stated. The cell-free broth was also maintained at a constant temperature (4, 28, 70, 100, and 120 °C) for 60 min and used for surface tension measurement. The effect of pH on surface tension was evaluated after adjustment of the broth pH to 2, 4, 6, 8, 10, and 12 with 6.0 M NaOH or HCl.

### Determination of surface tension and CMC of the biosurfactant

The surface tension was determined using a Sigma 700 tensiometer (KSV Instruments Ltd., Finland). The surface tension of Milli-Q water (72 mN/m) was used to calibrate the tensiometer. The measurements of surface tension were performed using the Du Noüy ring method. The analysis of surface tension were performed in triplicate on cell-free broth obtained by centrifuging the culture medium. CMC was determined by the surface tension obtained from frequent dilutions of the biosurfactant in Milli-Q water, until it reached a maximum surface tension in relation to concentration of surfactant molecules. The result of the CMC was obtained after stabilization of the concentration.

### Determination of biosurfactant toxicity

The lethality test with the brine shrimp was performed according to the method described by Meyer et al. (14). The biological assay was performed using the micro-crustacean *Artemia salina* incubated in 30 g/L of sea salt solution diluted in distilled water under 28°C at pH 8.0. Samples were processed in triplicate after 24 h incubation of larvae in a test containing 10 micro-crustacean *A. salina* in 5 mL per tube of solution. The following concentrations were used: 50, 100, 150, 300, 400, 500, and 600 mg/mL using the biosurfactant at the CMC and kept under artificial light. The calculation of nauplii mortality rate was carried out after 24 h. Mortality data were submitted to Probit analysis and lethal concentrations estimated using the POLO-PC software (LeOra Software Company, USA).

The phytotoxicity test was used to investigate the action of the biosurfactant on lettuce seeds (*Lactuca sativa* L.) and cabbage seeds (*Brassica oleracea* L.) (15). The disinfected seeds were placed in Petri plate on sterile filter paper and 5 mL of the isolated biosurfactant at the CMC in concentrations of 1, 5, and 50 mg/mL were added.

The determination was done after 120 h on the seed germination relative to root length and germination rate of the seeds, as follows: relative seed germination (%) = (number of seeds germinated in the extract/number of seeds germinated in control) × 100; relative root length (%) = (mean root length in the extract/mean root length in the control) × 100; germination index = [(% of seed germination) × (% of root growth)]/100%.

### Chemical composition of the biosurfactant

The protein concentration of the isolated biosurfactant was determined by the method of Lowry (16), using bovine serum albumin as standard. The carbohydrate content was determined by the method of phenol-sulfuric acid according to Dubois et al. (17) using D-glucose as a standard, while the total lipid content was measured by the method described by Folch et al. (18).

### Polyacrylamide gel electrophoresis

The molecular characterization of the proteins was carried out in polyacrylamide gel (12% w/v) under denaturing condition in the presence of sodium lauryl sulfate (SDS) and under reducing condition in the presence of 2-mercaptoethanol, according to the method described by Laemmli (19). Protein electrophoresis under acidic condition was performed according to Davis (20). The protein bands were subjected to staining with Coomassie Blue R-250, silver staining and Schiff staining. Bovine serum albumin (66 kDa), egg white albumin (45 kDa), carbonic anhydrase (29 kDa) and lysozyme (14.3 kDa) were used as molecular weight markers (Sigma-Aldrich, USA).

### Fourier transform infrared spectroscopy (FTIR)

To determine the infrared spectrum of the major functional groups of the isolated biosurfactant from *Streptomyces sp*. DPUA1559, it was submitted to a serial solubility test in different solvents in the ratio 1:1 (v/v), alternating the polarity of the solvents: hexane, dichloromethane, methanol, ethyl acetate and distilled water. The sample was analyzed by attenuated total reflection (ATR) technique in FTIR (ATR-FTIR). The spectrum was generated in the wavelength range of 4000 to 400 cm-1 using a Varian 640 IR FTIR spectrometer (Varian, Australia).

## Results and Discussion

### Experimental design through CCRD

A proper experimental design is based on the number of factors to be studied. The planning matrix obtained for the CCRD is shown in Table 2, where the variables (pH and temperature) in response to surface tension are presented.

**Table 2.** Planning matrix for central composite rotational design of experimental data for the biosurfactant produced by *Streptomyces sp*. DPUA1559 in culture medium after 96 h. pH: (X_1_); temperature °C: (X_2_); surface tension - mN/m: (Y).

Assay	pH	Temperature (°C)	Surface tension (mN/m)
1	8.40	27.0	30.40
2	8.40	29.0	28.00
3	8.60	27.0	29.38
4	8.60	29.0	27.47
5	8.36	28.0	30.73
6	8.64	28.0	28.85
7	8.50	26.6	28.68
8	8.50	29.4	26.95
9	8.50	28.0	25.47
10	8.50	28.0	25.96
11	8.50	28.0	25.59
12	8.50	28.0	24.34

Surface tension values pass through a central point indicating that the studied interval was suitable, when the surface tension reduction was used as a primary criterion for the production of the biosurfactant.

The CCRD was used to determine the production conditions of the surfactant agent from *Streptomyces sp*. DPUA1559 using ANOVA (Table 3). Parameters as experimental error, lack of fit, Fisher constant (F) and value of confidence level (p) are the main criteria for obtaining a statistical prediction model.

**Table 3.** ANOVA for the surface tension of the biosurfactant produced by *Streptomyces sp.* DPUA1559 in mineral medium containing 1% residual soybean oil after 96 h of fermentation.

Factor	Quadratic sum	Degrees of freedom	Quadratic mean	F	P
X_1_	2.22539	1	2.22539	4.59995	0.121308
${\text{X}}_{1}^{2}$	31.74989	1	31.74989	65.62788	0.003931
X_2_	5.67020	1	5.67020	11.72046	0.041735
${\text{X}}_{2}^{2}$	9.85354	1	9.85354	20.36753	0.020332
X_1_ * X_2_	0.05978	1	0.05978	0.12357	0.748437
Lack of fit	0.58603	3	0.19534	0.40378	0.762023
Experimental error	1.45136	3	0.48379		
Total	45.95987	11			

X_1_: pH; ${\text{X}}_{1}^{2}$: quadratic term of pH; X_2_: temperature (°C); ${\text{X}}_{2}^{2}$: quadratic term of temperature °C; X_1_ * X_2_: quadratic term of pH and temperature °C; R2 : 0.9557; R: 0.9187; F and P value in ANOVA test, where F_critical_ = 10.12 ${\text{X}}_{1}^{2}$.

The ANOVA indicates that the linear terms of temperature (X_2_) (X_2_) and quadratic term of pH and temperature are statistically significant, since the constant critical value of Fisher for these terms is less than the respective calculated values. This statistical significance is also observed when the respective values of confidence level were less than 0.05 (P<0.05). The linear terms of pH and the interaction between pH and temperature did not have statistical significance for the prediction model. The fit of the model and the relatively small value of the experimental error ensure that a good prediction model was obtained.

Figure 1 shows the Pareto diagram of the experimental assays, confirming what was observed through ANOVA (Table 3). The diagram indicates that the pH quadratic term is the most statistically significant term, followed in descending order by the quadratic term of temperature and linear term of temperature.

**Figure 1.** Effects of pH (X_1_ ${\text{X}}_{1}^{2}$) and temperature (X_2_ ${\text{X}}_{2}^{2}$) on biosurfactant surface tension.

Thus, only the individual values used were effective in lowering the surface tension. After these graphical and numerical analysis, a statistical prediction model was established for the operating range covered by the limits used in the CCRD. Therefore, to predict the surface tension, there is a model based on the regression coefficients obtained with the help of Table 1 (Equation 1):

(1) $$\text{Y=17653 - 81}{\text{.1X}}_{\text{2}}\text{+ 225}{\text{.5X}}_{1}^{2}+1.25{\text{X}}_{2}^{2}$$

The microorganism demonstrated great conditions for biosurfactant production in the temperature range 28 to 30°C for 96 h, evaluated with the soybean frying oil as the sole carbon source. The microorganism was able to reduce the surface tension of the medium in all assays.

The biosurfactant production was accompanied by surface tension measurements in the culture medium, which value decreased from 60 to 27.14 mN/m. The surface tension of the biosurfactant produced by *Streptomyces sp.* DPUA1559 were lower than the values of the surfactant produced by *Bacillus subtilis,* as reported by Mulligan (21) who observed a reduction of the surface tension to 27 mN/m. Lima e Silva et al. (22) showed that the surfactant from *Pseudomonas fluoresces* UCP1514 presented a surface tension of 31.68 mN/m when produced in corn steep liquor and burnt oil, and of 33.72 mN/m when produced in corn steep liquor and sunflower frying oil.

The aggregation of waste and by-products in media for the production of biosurfactants can minimize environmental impacts and reduce the production costs of biotechnological materials. Wastes and by-products have been used in several studies with different microorganisms to produce biosurfactants including fry waste of soybean oil, pineapple broth, burned sunflower oil, corn steep liquor, soybean oil, glycerol, ground nut oil refinery residue and soybean oil refinery residue, among others (2,23–27).

### Growth kinetics and biosurfactant production

After the establishment of the best conditions for cultivation by the CCRD, the growth kinetics and biosurfactant production were described.

Figure 2 shows the production kinetics of the biosurfactant from *Streptomyces sp*. DPUA1559 in mineral medium containing 1% residual soybean oil and 1% peptone during 120 h of cultivation. The microorganism exponential phase occurred in the first 24 h, corresponding to the adaptation phase to physical-chemical compositions of the culture medium. The biomass reached 1.26 g/L in this phase. The start of stationary growth phase and biosurfactant production occurred after 48 h. The biomass reached 4.81 g/L at 96 h. The maximum biomass concentration was around 5.02 g/L after 108 h of fermentation, followed by reduction of the surface tension, so the surface active properties of the biosurfactant were evidenced.

**Figure 2.** Kinetics of growth, pH, surface tension and biosurfactant production after 120 h of fermentation.

The pH of the fermentation medium varied between 6.8 and 7.7 in the first 24 h, and remained unchanged (between 8.0 and 8.7) during the rest of the fermentation period. This indicates that the microorganism adapts to the new substrate and promotes the biosynthesis of essential compounds to the growth, producing positive effects in reducing the surface tension and production stability (24,25 [Bibr B26]). According to Rufino et al. (8), each microorganism adapts to a specific pH for each type of biosurfactant to be produced.

After 120 h, the surface tension was reduced from 60 to 27 mN/m, although the surface tension values were less than 30 mN/m after 48 h. Silva et al. (28) have reported a reduction in the surface tension to 27.4 mN/m after 72 h of cultivation in the biosurfactant production by *P. aeruginosa* UCP0992, while Lima et al. (24) have observed a surface tension around 27.5 mN/m by a strain of *P. fluorescens*. The biosurfactant production by *Streptomyces sp*. DPUA1559 was observed in the stationary phase, after 96 h, with a yield of around 1.95 g/L. The full production was 2.24 g/L after 108 h of cultivation.

### Emulsification index with different hydrophobic compounds

The emulsification index was determined using the cell-free broth for different hydrophobic substrates: kerosene, motor oil, motor residual oil, diesel oil and vegetable oils (corn, canola, soybean and sunflower). The cell-free broth showed 38 and 40% emulsification of diesel and kerosene, respectively, while the emulsification index for motor oil and residual motor oil were respectively 89 and 95%. Silva et al. (28) reported an emulsification value of 53.7% for diesel, while a value of 50.2% was found for motor oil for the biosurfactant produced by *P. aeruginosa*.

Emulsification by the biosurfactant from *Streptomyces sp*. DPUA1559 showed 47, 41, 36, and 30% for corn oil, soybean oil, canola oil and sunflower oil, respectively. Rufino et al. (8) have observed an emulsification value for motor oil of 78%, while the corn oil was not effectively emulsified by the biosurfactant from *Candida lipolytica* UCP0998. The biosurfactant produced by *Streptomyces sp.* DPUA1559, in the conditions of this work, showed affinity for hydrophobic compounds tested, acting as surfactant agent and emulsifier.

### CMC of the biosurfactant

Figure 3 represents the CMC of the biosurfactant produced by *Streptomyces sp*. DPUA1559, which demonstrated a potential to reduce the surface tension from 70 to 33.76 mN/m, corresponding to a CMC of 10 mg/mL. Rufino et al. (8) reported a similar result for the biosurfactant produced by the yeast *C. lipolytica* UCP0998, whose CMC had a value of 10 mg/mL and a surface tension around 32 mN/m. Superior results of CMC have been obtained for biosurfactants isolated of *Streptomyces tendae* and *Streptomyces sp*. B3, whose values were respectively 36 mg/L and 110 mg/L (29,30). Gudina et al. (31) reported a CMC of 2.5 mg/mL of the biosurfactant produced by *Lactobacillus paracasei*.

**Figure 3.** Surface tension and critical micelle concentration of the biosurfactant after 96 h of fermentation.

A surface tension of 25.42 mN/m was reported by Chen et al. (32) for the biosurfactant produced from *B. licheniformis* TKU004 in a concentration of 350 mg/L, while Sobrinho et al. (33) has reported lower values of CMC for the biosurfactant of *C. sphaerica* UCP0995 of 0.08%.

### Stability of the biosurfactant

Purification accounts for up to 60% of the total production cost of biosurfactants. Because of economic considerations in the industry, most biosurfactants would require either whole-cell culture broths or crude preparations. Therefore, the application of the biosurfactant from *Streptomyces sp*. DPUA1559 in its crude form without prior costly extraction steps was investigated.

Figure 4 shows the influence of pH on surface tension of the cell-free broth from *Streptomyces sp*. DPUA1559 grown in soybean frying oil after 96 h of fermentation.

**Figure 4.** Influence of pH on the surface tension of the biosurfactant after 96 h of fermentation.

The results showed that the biosurfactant presented small changes in the values of surface tension when subjected to different pH values (4, 6, 8, 10) and it remained stable at pH 2 and 12 (30.23±0.04 mN/m). The graph shows that the lowest value of surface tension (27.14 mN/m) was obtained at pH 8, while the highest value was found at pH 2 (30.26 mN/m). Although the denaturation of protein compounds or increased ionization of the medium may cause the variation of the surface tension to extreme pH values (34), the graph shows that the biosurfactant had good surface activity in both acidic and basic media. The biosurfactant produced by *C. lipolytica* UCP0988 also presented a similar stability in the environmental conditions of pH (2–12) (8), while the biosurfactant from *C. sphaerica* UCP0995 was stable at a pH range from 2 to12 and with lower values of surface tension around 26 mN/m.

Figure 5 shows the effect of temperature on surface tension of the biosurfactant produced by *Streptomyces sp.* DPUA1559. The biomolecule showed resistance to the high and low temperatures studied, presenting thermal stability of surface tension. The surface tension was stable between 4–80°C. However, there was a slight increase (29.06 to 30.19 mN/m) of surface tension in a temperature range between 100–120°C. The surface tension in the temperature reported in this study are similar to those described by Khopade et al. (7) for the biosurfactant produced by *Streptomyces sp*. B3.

**Figure 5.** Influence of temperature on the surface tension of the biosurfactant after 96 h of fermentation.

Figure 6 illustrates the effect of different NaCl (%) concentrations on surface tension of the cell-free broth of *Streptomyces sp.* DPUA1559. The surface tension of the biosurfactant increased from 0% until 12%. The lowest value was 30.06 mN/m and the highest value was 33.38 mN/m. The biosurfactant surface tension was stable when subjected to high concentrations of NaCl, considering that concentrations above 2% of NaCl are enough to inhibit the activity of synthetic surfactants (35). Microbial surfactants synthesized by *C. lipolityca* UCP0988 and *C. sphaerica* UCP0995 were also stable in different concentrations of NaCl, confirming the results presented in this work (2,8).

**Figure 6.** Influence of different sodium chloride concentrations on the surface tension of the biosurfactant after 96 h of fermentation.

### Toxicity of the biosurfactant

The biosurfactant produced by *Streptomyces sp*. DPUA1559 showed no toxicity to the micro-crustacean *Artemia salina* at concentrations of 50, 100, and 150 g/mL based on its CMC of 10 mg/mL. The concentration of 600 mg/mL promoted 100% mortality. The lethal concentration was 300 g/mL, with 95% confidence interval, showing 40% of mortality. According to Saeki et al. (36), the biosurfactant JE1058BS produced by *Gordonia sp*. also demonstrated low toxicity to two species of marine larvae, *Bahia mysidopsis* (shrimp) and *Menidia beryllina* (fish). The biosurfactant produced by the yeast *C. sphaerica* UCP0995 showed no toxicity to the micro-crustacean *A. salina* (2).

Figure 7 represents the phytotoxicity promoted by the biosurfactant from *Streptomyces sp*. DPUA1559. The concentrations of the biosurfactant to the phytotoxicity tests of 1, 5, and 50 mg/mL did not display inhibitory effects on seed germination and root elongation after 5 days of incubation.

**Figure 7.** Effect of phytotoxicity of *Streptomyces sp*. biosurfactant on the seeds of lettuce and cabbage.

The germination indexes obtained for seeds of lettuce were 167, 110, and 92%, while for seeds of cabbage were 162, 126, and 100%, showing high germination, with good correlation between average elongation of root and germination index. The biosurfactants produced by *P. aeruginosa* UCP0992 promoted no toxicity to the seeds of *Lactuca sativa L*. and *Brassica oleracea L*. at concentrations similar to those reported in this work, as the lower concentrations of biosurfactant produced by *C. sphaerica* UCP0995 (2,28).

### Characterization of the biosurfactant

The biosurfactant produced by *Streptomyces sp*. DPUA1559 showed a chemical composition with 20% of proteins, 38% of carbohydrates and 12% of lipids. The protein portion marked with Periodic Acid-Schiff reagent was positive, indicating the presence of glycoproteins.

The biosurfactants isolated from several microorganisms can be lipids, glycolipids, lipopeptides and polysaccharide protein complexes (3). The biochemical composition of the biosurfactant probably depends on the substrates utilized in the culture medium. Rufino et al. (8) have reported that the biosurfactant isolated from *C. lipolytica* UCP0988 showed 50.0% of proteins, 8.0% of carbohydrates and 20.0% of lipids in the presence of refinery soybean oil. Other results were reported by Thavasi et al. (37), who showed that the biosurfactant of *Lactobacillus delbrueckii* has a composition 30.0% of carbohydrates and 70.0% of lipids. Luna et al. (2) obtained 15.0% of carbohydrate and 70.0% of lipid for the biosurfactant of *C. Sphaerica* UCP0995.

The molecular mass of the biosurfactant from *Streptomyces sp*. was around 14.3 kDa. The molecular characterization of the biosurfactant through the polyacrylamide gel showed a single protein band in the presence of denaturing and reducing conditions, revealing electrophoretic homogeneity. Moreover, the protein band exhibited acidic character.

Table 4 presents the main frequencies of the biosurfactant functional groups analyzed by ATR-FTIR. The spectral analysis of the solubilized biosurfactant in methanol presented intense bands characteristic of some functional groups. The spectra revealed a band at 3295 cm^−1^, indicating the presence of hydroxyl and a weak band at 2923 cm^−1^ related to the vibrations of axial deformation C-H of sp3 carbons. The low intensity of this signal indicates that there are no long chains of CH_2_ and CH_3_ groups in the molecule. Two bands at 1647 and 1559 cm^−1^ for amides were observed due to the angular deformation of NH_2_ and NH, known as the amide band II. Bands at 1454 and 1401 cm^−1^ of axial deformation of C=C of aromatic ring were observed and a broad band of medium intensity was observed in 1093 cm^−1^, characteristic of C-O axial deformation relative to primary alcohol. An intense band at 620 cm^−1^ indicates the frequency associated with the angular deformation for C=C, as well as the presence of halides such as chlorine, bromine or iodine.

**Table 4.** Characteristic spectral peaks analysis of biosurfactant produced by *Streptomyces sp.* DPUA1559 by ATR-FTIR.

Functional groups	Characteristic frequencies (cm^−1^)
Confirmed the presence of hydroxyl	3295
Weak bands related to the vibrations of axial deformation C-H of carbon sp^3^	2923
Amides and amides II observed due to angular deformation	1647 and 1559
Aromatic ring axial deformation of C=C	1454 and 1401
Broadband of axial intensity median of C-O	1093
Intense band	620

Infrared analysis indicated that the surfactant chemical structure is basically composed of peptides. The chemical profiles obtained by infrared analysis of the biotensoactive isolated and solubilized in water are identical, having only different polarities, basically composed of peptides. Although it presents amphiphilic characteristics, a detailed structural analysis of the biosurfactant is necessary to define its chemical structure.

The strain of *Streptomyces sp*. DPUA1559 demonstrated potential to produce surfactant molecules and emulsify in the presence of residual soybean oil. A prediction statistical model was important to establish the conditions of pH and temperature, optimizing the production of the biosurfactant. The molecule showed stability in extreme environmental conditions of pH, temperature and different salt concentrations. The biosurfactant was not toxic to micro-crustacean *Artemia salina*, and seeds of lettuce (*Lactuca sativa L*.) and cabbage (*Brassica oleracea L*.). The characterization showed a new surfactant with only one protein band having electrophoretic homogeneity and low molecular weight. The results are promising for a possible application of the biosurfactant in the industrial biotechnological area. Moreover, future investigations must be carried out in order to investigate its applications in the medical area.
